# Myricetin, a potent natural agent for treatment of diabetic skin damage by modulating TIMP/MMPs balance and oxidative stress

**DOI:** 10.18632/oncotarget.12330

**Published:** 2016-09-28

**Authors:** Zijian Wu, Xuemin Zheng, Min Gong, Ying Li

**Affiliations:** ^1^ Tianjin Key Laboratory of Food Biotechnology, College of Biotechnology and Food Science, Tianjin University of Commerce, Tianjin, China; ^2^ Tianjin Institute of Pharmaceutical Research, Tianjin, China; ^3^ Tianjin Neurological Institute, Tianjin Medical University General Hospital, Tianjin, China; ^4^ Department of Pharmacy, Tianjin Medical University, Tianjin, China; ^5^ Department of Oncology, University of Oxford, Oxford, UK

**Keywords:** myricetin, diabetic fibroblast, high glucose, oxidative stress, MMP

## Abstract

Foot ulceration is a major cause of morbidity in patients with diabetes, and abnormal peripheral neuropathy often results in hospitalization. Up-regulation of matrix metalloproteinases and down-regulation of tissue inhibitor of metalloproteinase 1 are noted to be distinctive biological functions of diabetic dermal fibroblasts. The aim of this study was to evaluate the biological effects of modified retinoids on diabetic fibroblasts. Myricetin, a natural compound, balances the TIMP1/MMP ratio and oxidative stress in diabetic fibroblasts. Our results indicate that myricetin significantly ameliorates the effects of diabetes on dermal fibroblasts. In addition, we found that the oxidative stress imbalance induced by a high glucose concentration plays an important role in the changes to dermal fibroblasts that occur in diabetes. Our findings support the hypothesis that myricetin has the potential to repair faulty skin function arising from diabetes.

## INTRODUCTION

Diabetic foot ulceration is a common and serious complication of diabetes that leads to 38,500 amputations each year [1]. It has been shown that reduced procollagen synthesis and increased levels of connective tissue-degrading matrix metalloproteinases (MMPs) are important factors in the early diagnosis of diabetic foot ulceration [2–5]. Tissue inhibitor of metalloproteinase-1 (TIMP1), an important component in balancing the TIMP1/MMP ratio [2, 6], is presumed to play an important role in the physiological characterization of diabetic fibroblasts and may be a biomarker for predicting the clinical morbidity of patients with diabetic foot ulceration [4]. Pustovrh et al. [7] found that in addition to regulating the TIMP1/MMP ratio, cellular oxidative stress affects MMP activities. González developed a relationship model of MMP activity and oxidative stress in diabetic rats, in which oxidative stress was shown to be involved in the developmental pathways of diabetic dermal fibroblasts [7]. More recently, it was found that high glucose levels in diabetic fibroblasts may be capable of inducing oxidative stress and mitochondrial dysfunction in neurons [8].

Myricetin is a bioflavonoid abundant in tea, berries, fruits, and vegetables (structure in Figure 1A) [9]. The history of myricetin in type 2 diabetes mellitus (T2DM) treatment and its complications is long-standing in southwestern China. It was reported that the anti-diabetic effectiveness of myricetin is due to its anti-inflammatory activity *in vitro* and in model animals [10]. Myricetin can *reduce* secretion of TNF-α and IL-1β in lipopolysaccharide (LPS)-stimulated RAW264.7 cells, and myricetin inhibited the production of IL-12 upon the down-regulation of transcription factor nuclear factor kappa-B (NF-κB) binding activity in RAW264.7 cells [11]. In addition, myricetin can decrease IL-1β-induced production of IL-6 in synovial cells, proving its anti-inflammatory activity, which was presumed to be associated with obesity-induced insulin resistance [12]. Liu et al. reported that injection of myricetin enhances insulin action in rats receiving fructose-rich chow [13]. Chang et al. found that dietary myricetin decreases body weight and improves the blood lipid profile in rats fed a high-fat diet [14]. Accumulating evidence suggests that myricetin may have the potential to alleviate obesity-induced insulin resistance through its anti-inflammatory activity and may be a promising therapeutic agent for treating T2DM. More recently, myricetin was found to modulate cellular oxidative stress, resulting in cytoprotective effects, by regulating the activities of antioxidant enzymes. Evidence indicated that the administration of myricetin is capable to ameliorate obesity-associated oxidative stress (glutathione peroxidase activity, total antioxidant capacity, and malondialdehyde) and inflammation (tumor necrosis factor-α) [15].

**Figure 1:** Effect of myricetin on the formation of active MMPs as determined by MMP zymography assays Legend (Panel **A**) Structure of myricetin. (Panel **B**). MMP zymography assay for MMP2 and MMP9. These results indicate that myricetin is capable of inhibiting the formation of MMPs in diabetic fibroblasts. Condition: Normal and diabetic fibroblasts were cultured in DMEM. The cells were routinely cultured in a humidified atmosphere at 37°C, 5% (v/v) CO_2_, and 95% (v/v) air and used for experiments between passages 3 and 5 (80% confluence). Culture media were assayed for MMP2 and MMP9 by casein and gelatin zymography.

The physiological properties of myricetin described in previous reports suggest that myricetin may help ameliorate complications of diabetes. To examine the effects of myricetin on diabetic skin damage, this study initially investigated the role that myricetin plays in balancing the MMP/TIMP1 ratio. Procollagen levels, which are important indicators of skin damage, are monitored upon myricetin administration. Finally, myricetin's function in regulating oxidative stress may be beneficial for understanding the mechanism by which myricetin suppresses skin damage in the presence of high glucose.

## RESULTS

### Effect of myricetin on diabetic fibroblasts

In this study, the effects of myricetin on diabetic dermal fibroblasts were investigated, including the levels of MMPs and TIMP1 in diabetic fibroblasts after four days of incubation with 3 μM myricetin, by using western blotting and qRT-PCR. Incubation of diabetic fibroblasts with myricetin significantly reduced the active MMP9 abundance, by 40% (*P* < 0.05) (Figure 1). In similarity, the levels of active MMP2 were also reduced by myricetin. On the basis of the data in Figure 2, the mRNA levels of MMP1, MMP2 and MMP9 were significantly down-regulated by myricetin, by 67%, 51% and 68% (*P* < 0.05), respectively. In contrast to the down-regulation of MMPs, myricetin induced a 72% increase in TIMP1 mRNA expression, as shown in Figure 2B (*P* < 0.05). Next, we examined the effects of myricetin on procollagen I and III expression levels using ELISA as these proteins are considered crucial to diabetic ulceration recovery in the clinic [16]. The protein levels of procollagen I and III in diabetic fibroblasts were increased after 4 days of treatment with myricetin. The levels of procollagen I and III increased by 103% and 53%, respectively, as shown in Figure 4. In addition, to study the effect of myricetin on oxidative stress on diabetic fibroblasts, two main cellular oxidative enzymes (catalase and superoxide dismutase) were analyzed. Following 4 days of incubation with 3 μM myricetin, the mRNAs of catalase and superoxide dismutase decreased by 50% and 64%, respectively (Figure 5, *P* < 0.05). Taken together, these results demonstrated the potency of myricetin in the treatment of diabetic foot ulceration and suggest that myricetin may achieve this end by balancing oxidative stress levels in diabetic fibroblasts.

**Figure 2:** Effects of myricetin on the ratio of TIMP1/MMPs in diabetic fibroblasts Legends (Panel **A)**. The normalized mRNA expression level of MMPs in diabetic fibroblasts in the presence of 3 μM myricetin. (Panel **B**). The normalized mRNA expression level of TIMPs in diabetic fibroblasts in the presence of 3 μM myricetin. (Panel **C**). The TIMP/MMP ratio in diabetic fibroblasts in the presence of 3 μM myricetin. These results show a decrease in the mRNA expression levels of MMP1, MMP2 and MMP9 in diabetic fibroblasts treated with 3 μM myricetin. After treatment, the mRNA expression level of MMP1 decreased by 67% (*P* < 0.05), the expression level of MMP2 decreased by 51% (*P* < 0.05), and the expression level of MMP9 decreased by 68% (*P* < 0.05). The mRNA expression level of TIMP1 was analyzed by qRT-PCR, and the data show that cells treated with myricetin had an mRNA expression increase of 72% (*P* < 0.05) compared with cells without myricetin incubation. Condition: The mRNA analysis kits for MMP1, MMP2 and MMP9 were supplied by the Shanghai Sangon Institute of Biology, and the mRNA analysis kit for TIMP1 was supplied by R&D Systems. The 2^−ΔΔCT^ method was used to analyze relative changes in gene expression.

**Figure 3:** Effects of high glucose on the molecular biomarkers of normal fibroblasts Legend These results suggest that high glucose increased MMP levels and decreased TIMP1 levels, *P* < 0.05. The presence of high glucose alters the ratio of MMPs to TIMP1, which is a standard diagnostic measure of diabetic foot ulceration. Condition: Normal dermal fibroblasts were cultured in DMEM media containing high glucose (16.7 mM) for four days. The mRNA expression levels of MMPs and TIMP1 were investigated by qRT-PCR, and the 2^−ΔΔCT^ method was used to analyze relative changes in gene expression.

**Figure 4:** Effects of myricetin on procollagen I and III Legend (top) Normalized protein abundance of procollagen I and III in diabetic fibroblasts treated with myricetin. (bottom) Western blotting analysis of procollagen I and III in diabetic fibroblasts treated with myricetin. Lane 1 shows the level of procollagen in the fibroblasts treated with myricetin. Lane 2 shows the level of procollagen in the fibroblasts not treated with myricetin. b-actin was employed as a control in this experiment. The procollagen I and III results suggest that myricetin induces higher expression levels of procollagen I and III in diabetic fibroblasts treated with myricetin. The images were digitized and quantified by scanning densitometry. Quantitative values for procollagen I and procollagen III were obtained and normalized against the normalization standards. The data show that myricetin induced increases in procollagen I (103%) and procollagen III (53%) in diabetic fibroblasts treated with myricetin, *P* < 0.05. Condition: Diabetic fibroblasts were incubated with 3 μM myricetin for four days in a humidified atmosphere at 37°C, 5% (v/v) CO_2_, and 95% (v/v) air and were used for experiments between passages 3 and 5 (80% confluence). The culture media were assayed for procollagen I and procollagen III by western blotting.

**Figure 5:** Effects of myricetin on catalase and superoxide dismutase in oxidative stress Legend (Panel A). Myricetin induced a 50% decrease in the mRNA expression level of catalase in diabetic fibroblasts. Panel B. Myricetin induced a 64% decrease in the mRNA expression level of superoxide dismutase in diabetic fibroblasts. These data indicate that the mRNA levels of both catalase and superoxide dismutase decrease in the presence of 3 μM myricetin. Catalase and superoxide dismutase are involved in the induction of cellular oxidative stress, which is attributed to a rise in MMP expression and activation. Condition: The cells were incubated with 3 μM myricetin for four days, and then the expression levels of catalase and superoxide dismutase were examined by qRT-PCR. The 2^−ΔΔCT^ method was used to analyze relative changes in gene expression.

### Effects of high glucose on molecular biomarkers in normal fibroblasts

We were also interested in investigating the role of high glucose in normal fibroblasts and determining whether the presence of high glucose can alter molecular biomarkers, including MMPs and TIMP1. In this study, dermal fibroblasts from healthy females were cultured in a medium containing high glucose (16.7 mM, a similar level to that used in diabetic subjects). Then, the mRNA expression levels of several biomarkers [e.g., MMP1, MMP2, MMP9 and TIMP1] were analyzed using qRT-PCR and compared with those of biomarkers from normal fibroblasts. The results showed that the mRNA levels of MMP1, MMP2 and MMP9 from normal fibroblasts in high-glucose media were significantly up-regulated (Figure 3). The increased expression of MMPs in response to high glucose coincided with a reduction in TIMP1 levels. The results suggest that fibroblasts cultured in a high-glucose medium exhibit biological characteristics similar to those of diabetic fibroblasts. This finding is useful for efficiently carrying out in-vitro drug screening.

## DISCUSSION

In diabetes, the lifetime risk of developing a foot ulcer is estimated to be 5%–15%. Approaches aimed at reducing the risk of ulceration or improving healing rates are urgently required for more severe diabetes. The causes of ulceration in diabetic patients are multifactorial but may be accelerated by changes in the structure and function of the skin, including impaired fibroblast proliferation, decreased collagen synthesis and increased matrix metalloproteinase (MMP) expression [17]. Increased elaboration of activated MMPs is thought to precede changes in skin structure, which is then followed by a reduction in collagen synthesis and widespread collagen destruction [18–20]. Pro-MMP2 and pro-MMP3 levels are reportedly increased in the fibroblasts of diabetic patients [21]. Recently, catalase and superoxide dismutase were considered to be involved in oxidative stress induction because oxidative stress presumably contributes to the up-regulation of MMPs [7]

The biological effects of myricetin on diabetic fibroblasts were initiated to investigate the TIMP1/MMP ratio, the main indicator for evaluating the progress of diabetic ulceration. Figure 2C clearly demonstrates a significant increase in the TIMP1/MMP ratio following myricetin treatment. Interestingly, the incubation of high glucose in normal fibroblasts induced a decrease in the TIMP1 expression level and rise on MMPs, as shown in Figure 3. It is hypothesized that the oxidative stress induced by high glucose concentrations may contribute to oxidative stress imbalance and morbidity in patients with diabetes as high glucose levels may induce oxidative stress and apoptosis in the neurons of patients with diabetes [22–24]. The effects of myricetin on type I and III procollagen were also investigated. Myricetin stimulated procollagen synthesis, which was proposed that myricetin may utilize signaling mediation through the JNK pathway, a potent inducer of procollagen production [25]. In addition, myricetin down-regulated the expression of catalase and superoxide dismutase—the two main enzymes involved in the induction of cellular oxidative stress, those play important role in the pathogenesis of type 2 diabetes mellitus and its complications [26].

In conclusion, myricetin seems to possess the necessary potency to reverse the activation of connective tissue-degrading MMPs, increase the procollagen abundance and ameliorate the oxidative stress in high-risk patients, as showed in Figure 6. Myricetin treatment may be beneficial in preventing chronic diabetic foot ulceration in the clinic. The results of this study may provide a basic framework for skin damage caused by T2DM.

**Figure 6:** Functions of myricetin on MMPs/TIMP1 regulation and oxidative stress Myricetin is capable to possess the necessary potency to reverse the activation of connective tissue-degrading MMPs, increase the procollagen abundance and ameliorate the oxidative stress in high-risk patients.

## MATERIALS AND METHODS

### Materials

The diabetics fibroblasts were provided by Dr. Ying Li (donation from female T2DM patient, age 59) originated from female diabetes patient. The cell line was incubated in a 24-well plate containing 260 μl of Ca^2+^ (50 μM) supplemented MCDB-153 medium per well at 37°C in an atmosphere of 95% air and 5% CO_2_ for 8 days. Culture media were collected and replaced every second day. Healthy human dermal fibroblasts supplied by the Institute of Biochemistry and Cell Biology, China Academy of Sciences (Shanghai, China) were cultured in Dulbecco minimal Eagle's medium (DMEM), which contains a high glucose concentration (16.7 mM). The cells were routinely cultured in a humidified atmosphere at 37°C, 5% CO_2_, and 95% air, and cells between passages 3 and 5 (80% confluence) were used for experiments. The participation of human subjects in this project was approved by the appropriate local ethics committees, and all subjects provided written informed consent prior to their inclusion in the study. Myricetin (Figure 1A) was purchased from Sigma-Aldrich Chemical Company (CAS 529-44-2, Mw 318.24, Shanghai, China)

### Quantitative real time PCR (qRT-PCR)

mRNA analytical kits for detecting MMP1, MMP2, MMP9, TIMP1, catalase and superoxide dismutase were purchased from the Shanghai Sangon Institute of Biology (Shanghai, China), and the 2^−ΔΔCT^ method was used to analyze relative changes in gene expression.

### MMP assays

Medium from fibroblast cells was assayed for the levels of MMP2 and MMP9 by casein and gelatin zymography. Zymographic images were digitized and quantified by scanning densitometry. Quantitative values for the expression levels of MMP2 and MMP9 protein were obtained and normalized against MMP normalization standards.

### ELISA assay for TIMP1

Culture media were assayed for the abundance of TIMP1 by enzyme-linked immunosorbent assay (ELISA), using a commercially available assay kit (R&D Systems, Minneapolis, US).

### Western blotting

Procollagen type I and III protein expression levels were detected by Western blotting. Antibodies were purchased from Santa Cruz Biotechnology Inc (California, US) and used according to the manufacturer's protocols.

### Statistical analysis

Student's *t*-test and ANOVA was employed for analyzing data. Unless otherwise stated, the results were reported as the mean ± standard error. *P* values less than 0.05 were considered significant.
